The article "Body Fat Evaluation in Male Athletes from Combat Sports by Comparing Anthropometric, Bioimpedance, and Dual-Energy X-Ray Absorptiometry Measurements" was published in 2022. Journal: Biomed Res Int.

# Body Fat Evaluation in Male Athletes from Combat Sports by Comparing Anthropometric, Bioimpedance, and Dual-Energy X-Ray Absorptiometry Measurements

**DOI:** 10.1155/2022/3456958

**Published:** 2022-09-05

**Authors:** Marko Dimitrijevic, Verica Paunovic, Vladimir Zivkovic, Sergey Bolevich, Vladimir Jakovljevic

**Affiliations:** ^1^Department of Physiology, Faculty of Medical Sciences, University of Kragujevac, Svetozara Markovica, 69 Kragujevac, Serbia; ^2^Institute of Microbiology and Immunology, Faculty of Medicine, University of Belgrade, Dr Subotica 1, Belgrade, Serbia; ^3^Department of Human Pathology, First Moscow State Medical University I.M., Bol'shaya Pirogovskaya Ulitsa, 2 Sechenov, Russia; ^4^First Moscow State Medical University I.M., Bol'shaya Pirogovskaya Ulitsa, 2 Sechenov, Russia

## Abstract

Multiple anthropometric equations have been developed aiming to provide accurate and affordable assessment of body fat composition in male athletes. This study examined correlations of values obtained from seventeen different anthropometric equations to DXA as well as BIA and DXA values. Male athletes (*n* = 101) from three different combat sports, wrestling (*n* = 33), judo (*n* = 35), and kickboxing (*n* = 33), with an average age of 20.9 ± 4.2 were included. Body fat percentage was estimated using anthropometry, BIA, and DXA. Correlations between anthropometric methods and DXA, as well as BIA and DXA, were determined using Spearman's rank correlation. Sixteen out of seventeen estimates of body fat percentages using existing anthropometric equations showed strong positive correlation with the values derived from DXA measurements (*r* = 0.569 − 0.909). The highest correlation was observed using the equation derived by Yuhasz, *r* = 0.909, followed by the equations from Oliver et al., Evans et al., Faulkner, and Thorland et al. (*r* ≈ 0.9). Statistical analysis of body fat percentages from DXA and BIA measurements also showed high positive correlation (*r* = 0.710). Correlation of seventeen anthropometric equations with BIA and DXA methods revealed that equations by Yuhasz, Oliver et al., Evans et al., Faulkner, and Thorland et al. are suitable alternative for assessing body fat percentage among male athletes from combat sports, showing even stronger correlation than BIA method.

## 1. Introduction

Body composition of athletes has a paramount effect on physiology and physical performance and provides information on the overall health [1]. The body fat percentage (%BF) is an important component of the athlete's body since adipose tissue has a complex effect on the health in general [2]. Adipose tissue is a vital endocrine organ [3], but both low and high %BF pose a threat for athlete's performance [4]. Previous studies have showed that high levels of body fat have negative impact on aerobic and anaerobic capacity of soccer players [5] and present serious cardiometabolic risk [6]. On the other hand, low body fat percentage (less than recommended 12%) is associated with low energy availability and both micro- and macronutrient deficiency in female gymnasts, thus posing threat to athlete's health and performance [7].

The article "Body Fat Evaluation in Male Athletes from Combat Sports by Comparing Anthropometric, Bioimpedance, and Dual-Energy X-Ray Absorptiometry Measurements" was published in 2022. Journal: Biomed Res Int.

Body composition can be quantified at multiple levels: atomic level (measurement of carbon, calcium, potassium, and hydrogen quantity), molecular level (assessment of amounts of water, protein, and fat), cellular level (assessment of extracellular fluid and body cell mass), and at the tissue level (determination of amounts and distributions of adipose, skeletal, and muscle tissues) [8]. Accurate quantification of body composition has been the subject of intense research for decades. This scientific effort resulted in developing a large number of quantification methods, which include direct (cadaver dissection) and an array of indirect methods [1]. Indirect assessment of body properties, such as density, distribution of skeletal muscle, and adipose tissues, is performed using computed X-ray tomography (CT), magnetic resonance imaging (MRI), and dual-energy X-ray absorptiometry (DXA) [1]. These methods, referred to as second level of validity methods, are complex and performed in highly specialized facilities and require substantial financial means. Accordingly, less complex indirect methods of body composition assessment (third level of validity methods) such as bioelectrical impedance analysis (BIA) and anthropometry have been developed as more accessible to wider user population to provide an estimate of body composition [8]. However, to be applied accurately for a specific population, these methods have to be validated against the direct or second level of validity methods such as DXA. Moreover, BIA and anthropometry have larger predictive errors than the direct and second level of validity methods and are significantly affected by the sample population specificity [8]. However, they are still often considered as a suitable replacement and used among sports coaches and experts in practice. In circumstances such as travel to preparation camps or competition, these lower cost and portable methods are widely used due to their practicality, portability of measuring devices, and the fact that they do not require highly skilled staff to perform the measurements.

Wrestling, judo, and kickboxing are classified as weight-sensitive sports, in which athletes tend to undergo extreme dieting associated with extreme dehydration in order to reduce body mass, more specifically %BF, aiming to be moved to a lower weight category [1]. Therefore, regular measurements of body composition for this specific athlete population are extremely important. Taking into account that previous studies have already established that anthropometric equations developed for general nonathlete population are not applicable for professionals [9] and that the ones developed for athletes are highly specific for the specific sport [9–11], there is a pressing need to validate existing anthropometric equations, developed for both general and specific athlete population, and BIA against a reference gold standard method DXA in general athlete population.

The article "Body Fat Evaluation in Male Athletes from Combat Sports by Comparing Anthropometric, Bioimpedance, and Dual-Energy X-Ray Absorptiometry Measurements" was published in 2022. Journal: Biomed Res Int.

The aim of this study was to explore the correlations of different developed anthropometric equations with DXA measurements as well as the correlations of BIA with DXA measurements in determining the percentage of body fat in male athletes.

## 2. Materials and Methods

### 2.1. Study Design

The study was designed as a cross-sectional observational analysis of competitive, successful, and world-class elite male athletes competing in wrestling, judo, and kickboxing [12]. All participants were assessed within three days in 2021. The study was approved by the Ethical Committee of the Faculty of Medical Sciences, University of Kragujevac (License number 01-14980) in accordance with the current national and international laws and regulations controlling the use of human participants (Declaration of Helsinki II).

### 2.2. Participants

Analyzed population sample consisted of 101 athletes (*N* = 101), 17-33 years of age, recruited from three different combat sports: wrestling (*n* = 33), judo (*n* = 35), and kickboxing (*n* = 33). Recruited athletes showcased similarities related to their body composition, preparation, and monitoring prior to attending and during competitions. Inclusion criteria consisted of athletes who fulfilled classification criteria for “eliteness” or expertise defined by Swann et al. [12]. In brief, athletes who were competing for more than 3 years at national and/or international level and did not have any long training breaks or any rest caused by an injury or any other factor within the last six months were included in the study. After detailed explanation of the procedure and study goals, athletes who decided to participate in this study signed a voluntary consent document.

### 2.3. Procedures

Participants were divided into three groups and scheduled to come to DXA cabinet room at the Department of Orthopedy, Clinical Centre of Vojvodina, Novi Sad, between 9 and 10 h in the morning for three consecutive days. They were instructed to follow standard food and fluid intake so they are in a rested, overnight fasted (at least 8 h), and hydrated state before testing. Moreover, they were asked not to perform any physical activity prior to their evaluations and to bring light cotton clothing. Complete testing of every individual athlete was conducted on the same day. Participants were evaluated by BIA, anthropometric measurement, and a whole body DXA scan, respectfully. All the equipment was calibrated each morning on the day of analysis prior to measurements.

The article "Body Fat Evaluation in Male Athletes from Combat Sports by Comparing Anthropometric, Bioimpedance, and Dual-Energy X-Ray Absorptiometry Measurements" was published in 2022. Journal: Biomed Res Int.

### 2.4. Anthropometric Measurements

Anthropometric measurement of skinfolds, circumferences, and joint bone diameters was conducted according to ISAK guidelines and recommendations [13]. Body weight was measured during BIA test. After BIA analysis was completed, anthropometric measurements of body height, skinfolds, circumferences, and joint diameters were conducted. An anthropometrist (>10 years of experience) was recruited to perform anthropometric measurement.

Firstly, skinfolds (subscapular, midaxillary, chest (pectoral), abdominal, biceps, triceps, suprailiac, supraspinale, quadriceps, and medial calf) were located and labeled with a marker as determined by ISAK guidelines [13]. Then, skinfolds were measured using Harpenden caliper (HSB-BI, HaB Direct, UK). The caliper has measuring range of 0-80 mm (caliper needle is made to go four full circles around a dial scale graduated from 0 to 20 mm), measuring pressure of 10 g/mm^2^, and reading accuracy of 0.2 mm. The height was measured using roll-up measuring tape (SECA, Germany) with measuring range of 0-220 cm (1 mm graduation). Circumferences were determined using a flexible steel tape calibrated in centimeters with millimeter graduations (Lufkin metal tape). Small sliding caliper (Rosscraft) was used to measure biepicondylar breadths of humeri and femurs. The instrument has a branch length of 10 cm, an application face width of 1.5 cm, and an accuracy of 0.05 cm.

Seventeen anthropometric methods [9–11, 14–21] developed for different male athlete populations through regression analysis were used in this study (Table 1). Selected anthropometric equations were developed for either a specific or general sport population, based on skinfold measurements alone or skinfold measurements combined with some basic anthropometric/descriptive features such as age, body height and weight, and body mass index. Moreover, equations selected for our study presented the highest multiple correlation coefficients between a dependent variable and a group of independent variables (*R*), or the largest variance in dependent variable by using independent variables (*R*^2^) (depending on what was reported in a particular study, *R* or *R*^2^), when correlated with referent methods. Furthermore, the Siri equation was used to convert body density to body fat percentage in cases where anthropometric equations estimated only body density [22]. The test-retest reliability of anthropometric measurement was determined using the method of technical measurement error (TEM) of an evaluator, where a deviation of up to 7.5% for skinfolds and up to 1.5% for other anthropometric measures was considered acceptable. The calculation of the TEM was carried out according to the recommendations by Norton [23].

The article "Body Fat Evaluation in Male Athletes from Combat Sports by Comparing Anthropometric, Bioimpedance, and Dual-Energy X-Ray Absorptiometry Measurements" was published in 2022. Journal: Biomed Res Int.

### 2.5. Bioelectrical Impedance Analysis (BIA)

Upon arrival, participants were subjected to the bioelectrical impedance analysis (BIA) for measurement of the body fat percentage and body weight as described in our previous study [24]. The measurement was conducted according to the manufacturer's instructions for model InBody 230 using BIA pretest guidelines [24, 25]. In brief, prior to measurement, every participant had their palms and soles wiped with a tissue containing electrolyte solution. Next, the participants stood on the scales with their soles in contact with the foot electrodes for weight measurement. Then, age, sex, and height were entered into the instrument. The participants were then instructed to firmly grasp hand grips by placing their thumb and fingers on the designated locations, and the impedance was measured. The measurements were conducted by an experienced InBody 230 operator.

### 2.6. Dual-Energy X-Ray Absorptiometry (DXA) Scanning

DXA scanning was performed for each participant on Lunar iDXA scanner (GE Healthcare, UK) according to the current guidelines for best practice [26]. Quality control was assured by calibration procedure according to the manufacturer's instructions. In brief, the apparatus was calibrated every morning, or whenever the temperature in the room changed for 5°C, by using appropriate calibration blocks (three for bone density and three for whole body measurements). The participants wearing light cotton clothing were positioned in a stationary, supine position on the scanning table with keeping hands in the hip level and feet slightly apart. Upon taking a proper position, the scan was initiated and lasted for about 6 minutes. All the measurements and calibration procedures were performed by an experienced, certified DXA technician to ensure consistency in measurement protocols. Technical error of DXA scanner measurement was 3%. Scans were analyzed using enCORE software V17 (GE Healthcare, UK).

### 2.7. Statistical Analysis

Statistical analysis was conducted using SPSS statistical program, package version 26 (IBM SPSS Statistics for Windows, Armonk NY: IBM Corp; 2018). Assessment of linearity for model validity, outliers, and data normality distribution was performed using scatter plot graph, Q-Q plot, histogram, skewness and kurtosis, and the Kolmogorov-Smirnov test. Based on the information obtained by these tests, assessment of the correlation of estimates obtained using anthropometric equations and BIA measurement was conducted using Spearman's rank correlation (*r*), where values of *r* = 0.0–0.09 were considered trivial, *r* = 0.10–0.29 small, *r* = 0.30–0.49 moderate, *r* = 0.50–0.69 high, *r* = 0.70–0.89 very high, *r* = 0.90–0.99 almost perfect, and *r* = 1 perfect correlation [27]. Descriptive data was presented through means and standard deviations (mean ± SD). Statistical significance (*p* values) was set at 0.05. Confidence interval was set at 95%. Graphs were created using GraphPad Prism 7.04.

The article "Body Fat Evaluation in Male Athletes from Combat Sports by Comparing Anthropometric, Bioimpedance, and Dual-Energy X-Ray Absorptiometry Measurements" was published in 2022. Journal: Biomed Res Int.

## 3. Results

Characteristics of participants are presented in Table 2. Anthropometric measurements of skinfolds were converted into body fat percentage (%BF) using seventeen equations listed in Table 1.

Sixteen out of seventeen estimates of %BF showed strong positive correlation (*r* = 0.569 − 0.909) with the values derived from DXA measurements (Table 3 and Figure 1). The highest correlation (*r* = 0.909) was observed using the equation derived by Yuhasz et al. [14]. Nevertheless, the equations from other authors (Oliver et al., Evans et al., Faulkner, and Thorland et al. [10, 16, 18, 20]) showed very similar correlation coefficients (*r* values over 0.9); only the *r* value obtained from the equation by Zuti and Golding was smaller than 0.6 [15]. Statistical significance of all anthropometric equations applied was high with *p* < 0.001. In addition, the 95% confidence intervals showed wide ranges and overlap (Table 4).

Statistical analysis of the %BF estimates obtained from DXA and BIA measurements also showed high positive correlation with high statistical significance (*r* = 0.710, *p* < 001) (Table 5).

## 4. Discussion

The aim of this study was to compare the accuracy of body fat assessment by anthropometric measurements and BIA, using DXA as a criterion (also referred to as one of the “gold standard” methods), in male athletes from combat sports. Furthermore, the ultimate objective was to uncover the most precise existing anthropometric equation developed using specific anatomical landmarks for skinfolds, circumferences, joint diameters, and basic physical measurements and characteristics (such as weight, height, age, BMI, and WHR) applicable to the male athletes from combat sports. Correlation results of seventeen anthropometric equations with BIA and DXA methods revealed that equations by Yuhasz, Oliver et al., Evans et al., Faulkner, and Thorland et al. showed very high correlation with the values obtained by DXA method, even stronger than the BIA values. Therefore, these equations are considered as a suitable alternative for assessing body fat percentage in male athletes from combat sports.

The article "Body Fat Evaluation in Male Athletes from Combat Sports by Comparing Anthropometric, Bioimpedance, and Dual-Energy X-Ray Absorptiometry Measurements" was published in 2022. Journal: Biomed Res Int.

To date, many studies proposed novel anthropometric measurements and equations for body fat assessment. However, these methods are mostly population-specific developed for a particular sports or nation-specific, i.e., applicable to anthropometric characteristics of a particular nation studied [10, 17, 21, 28–33]. Moreover, this myriad of methods may cause bewilderment in coaches and sports experts in selecting a correct method for their athletes. Therefore, inadequate choice of method may lead to significantly inaccurate assessment of body fat, thus affecting management of body fat regulation, especially in weight-sensitive sports.

Prior to choosing the adequate anthropometric measurement for their athletes, the coaches/sports experts should take into account gender, race, age, nation, condition and competition level, protocols for skinfolds, and other anthropometric measurements as well as other specific characteristics of athlete population used for the development of the chosen method. Even if all the criteria are met, it is not a guarantee that the selected method would be accurate enough for their particular athletes, most likely affected by slight or more significant differences between the athlete sample used for anthropometric method development and their athletes. This suggests that practically every coach should develop an equation specific for his team which is cumbersome and time-consuming task. Therefore, for athlete body composition assessment, DXA is still the “gold standard” method, while BIA has been the preferred field method over anthropometry. However, anthropometric measurements still have significant advantages over DXA and BIA, since anthropometric instruments take up less space, are not performed in specialized facilities, do not have complicated electronics prone to damage, and cannot be affected by potential physiological oscillations in human body caused by air travel or change of time zone. Moreover, anthropometric measurements do not require strict preparation protocols prior to testing (BIA) or highly skilled operator to perform the measurement (DXA). Taking into account all the above, this study was aimed at assessing which of the existing anthropometric measurements and equations has the correlation coefficient closest to both BIA and DXA, which are second-level validity referent methods, and thus be suggested as an accurate alternative in the field practice. To the best of our knowledge, more than hundreds of anthropometric methods and equations have been developed to date. In this study, estimates obtained by using seventeen well-known methods/equations used for a number of decades were correlated with DXA. Sixteen estimates of %BF showed strong positive correlation with the values derived from DXA measurements. This is an intriguing finding considering that the anthropometric methods/equations analyzed in this study have been diverse. They were developed over more than a fifty-year span either for athletes from different sports or on more general athlete population, using different references and criterion methods or applying different models for body composition assessment. Therefore, greater variability in correlation coefficients with DXA method was expected. Surprisingly, the majority of the correlation coefficients of anthropometric measurements were higher than the correlation coefficient of BIA with DXA method. However, considering relatively wide ranges and overlap between the 95% confidence intervals, the comparison between the correlation coefficients should be done with special attention.

The article "Body Fat Evaluation in Male Athletes from Combat Sports by Comparing Anthropometric, Bioimpedance, and Dual-Energy X-Ray Absorptiometry Measurements" was published in 2022. Journal: Biomed Res Int.

The study has several limitations. For example, even though widely used as a reference method in estimation of body fat content, DXA method is known to have moderate precision and accuracy in assessing percentage of body fat [34]. Also, DXA results can vary from different machines and software [35]. Furthermore, readings from BIA apparatus are generated by proprietary prediction equations unknown to users. Even though this study included relatively large number of participants, all of them were young Caucasians; therefore, the future studies are required to validate our findings on population of different ethnicity or even gender. Despite the described shortcomings, the study has been performed using wide variety of methods to estimate body fat percentage in a population of elite athletes. Most importantly, the presented findings have shown that anthropometry is an accessible and a suitable alternative to DXA and BIA methods for assessing %BF in combat sports such as wrestling, judo, and kickboxing.

## 5. Conclusions

The aim of this study was to find which of the existing anthropometric equations can be used as an accurate yet affordable replacement for BIA and more importantly DXA method in male athletes from combat sports. The highest correlation was observed using the equation derived by Yuhasz; however, the equations from Oliver et al., Evans et al., Faulkner, and Thorland et al. showed very similar correlation coefficients. Moreover, all the equations with exception of Zuti and Golding seem to be more reliable than BIA method. Therefore, anthropometric equations derived by Yuhasz [14], Oliver et al. [10], Evans et al. [20], Faulkner [18], and Thorland et al. [16] appear to be more affordable alternatives to DXA and BIA to which coaches and sports experts can resort to when these more complex methods are not a suitable option.

The article "Body Fat Evaluation in Male Athletes from Combat Sports by Comparing Anthropometric, Bioimpedance, and Dual-Energy X-Ray Absorptiometry Measurements" was published in 2022. Journal: Biomed Res Int.

## Figures and Tables

**Figure 1:** Graphs representing correlation between existing anthropometric equations and DXA-derived estimates of assessing body fat percentage of in male athletes from combat sports.

**Table 1:** Selected existing anthropometric methods and equations developed for assessing body fat in different male athletes and general and specific populations.

Author(s)/method	Anthropometric equation
Yuhasz [14]	Equation using 6 skinfolds: %BF = 3.64 + (0.097 (Ch + Tr + Sb + Si + ab + Th))
Faulkner [33]	Equation using 4 skinfolds. Today considered a modified Yuhasz method: %BF = 5.783 + (0.153 (Tr + Sb + Si + ab))
Forsyth and Sinning 1 [9]	Equation using 2 skinfolds (equation no. 2a): BD = 1.103 − (0.00168 × Sb) − (0.00127 × ab)
Forsyth and Sinning 2 [9]	Equation using 4 skinfolds (equation no. 2b): BD = 1.10647 − (0.00162 × Sb) − (0.00144 × ab) − (0.00077 × Tr) + (0.00071 × ma)
Forsyth and Sinning 3 [9]	Equation using 2 skinfolds and height (equation no. 3a): BD = 1.02415 − (0.00169 × Sb) + (0.00444 × Ht)–(0.00130 × ab)
Forsyth and Sinning 4 [9]	Equation using 4 skinfolds and height (equation no. 3b): BD = 1.03316 − (0.00164 × Sb) + (0.00410 × Ht)–(0.00144 × ab)–(0.00069 × Tr) + (0.00062 × ma)
White et al. [11]	Equation using 2 skinfolds: BD = 1.0958 − (0.00088 × Si) − (0.0006 × Th)
Thorland et al. 1 [16]	Equation using 7 skinfold: BD = 1.1091 − (0.00052 (Tr + Sb + ma + Si + ab + Th + ca)) + (0.00000032 (Tr + Sb + ma + Si + ab + Th + ca)^2^)
Thorland et al. 2 [16]	Equation using 3 skinfolds: BD = 1.1136 − (0.00154 (Tr + Sb + ma)) + (0.00000516 (Tr + Sb + ma)^2^)
Withers et al. [19]	Equation using 7 skinfolds, not fully published in the original 1987 paper by Withers et al., but can be found in Reilly et al. study derived from Withers et al. data. BD = 1.0988 − (0.0004 (Tr + Sb + Bc + Sp + ab + Th + ca))
Evans et al. 1 [20]	Equation using 7 skinfolds, gender and race: %BF = 10.566 + (0.12077 (Sb + Tr + Ch + ma + Si + ab + Th))–(8.057 × gender) − (2.545 × race)
Evans et al. 2 [20]	Equation using 3 skinfolds, gender and race: %BF = 8.997 + (0.24658 (ab + Th + Tr))–(6.343 × gender)–(1.998 × race)
Oliver et al. [10]	Equation using 7 skinfolds (equation model number 3): %BF = 3.53 + (0.132 (Ch + Tr + Sb + ma + Si + ab + Th))
Reilly et al. [17]	Equation using 4 skinfolds: %BF = 5.174 + (0.124 × Th) + (0.147 × ab) + (0.196 × Tr) + (0.13 × ca)
Civar et al. [21]	Equation using 3 skinfolds and weight: %BF = (0.432 × Tr) + (0.193 × ab) + (0.364 × Bc) + (0.077 × Wt)–0.891
Stewart and Hannan [30]	Equation using 2 skinfolds and weight. This equation estimates body fat in grams, which are then converted into body fat percentage for BIA comparison: BFM = (331.5 × ab) + (356.2 × Th) + (111.9 × Wt) − 9108
Zuti and Golding [15]	BD = 1.0806 − (0.001187 × WC) − (0.001076 × Ch) + (0.015306 × WD)

Ht: height; Wt: weight; BD: body density; %BF: body fat percentage; BFM: body fat mass in grams; Tr: triceps skinfold; Ma: midaxillary skinfold; Sb: subscapular skinfold; Ab: abdominal skinfold; Si: suprailiac skinfold; Sp: supraspinale skinfold; Th: quadriceps skinfold; Ca: calf skinfold (medial calf); Ch: chest skinfold; Bc: biceps skinfold; gender: *mаn* = 1, woman = 0; race: African American = 1, Caucasian = 0; WC: waist circumference; WD: wrist diameter.

The article "Body Fat Evaluation in Male Athletes from Combat Sports by Comparing Anthropometric, Bioimpedance, and Dual-Energy X-Ray Absorptiometry Measurements" was published in 2022. Journal: Biomed Res Int.

**Table 2:** Athlete descriptive characteristics.

Variable	Wrestlers	Judokas	Kickboxers	Total
	*X* ± SD	*X* ± SD	*X* ± SD	*X* ± SD
Age (years)	18.6 ± 1.9	23.9 ± 4.2	22.8 ± 5.4	20.9 ± 4.2
Height (cm)	177.2 ± 8.6	178.1 ± 7.1	183.8 ± 6	179.8 ± 7.8
Weight (kg)	77.7 ± 15.5	79.0 ± 15.9	83.0 ± 13.3	80, 0 ± 14.0
BMI (kg/m^2^)	24.6 ± 3.3	24.8 ± 3.4	24.5 ± 3.3	24.0 ± 3.3
WHR (cm^2^)	0.85 ± 0.06	0.85 ± 0.6	0.84 ± 0.07	0.85 ± 0.06
%BF_BIA_	11.4 ± 4.9	11.0 ± 5.5	11.3 ± 5.3	11.2 ± 5.2
%BF_DXA_	16.1 ± 5.1	16.5 ± 6.1	18.2 ± 5.6	17.0 ± 5.7

*X*: mean; SD: standard deviation; BMI: body mass index; WHR: waste-to-hip ratio; %BF_BIA_: body fat estimated with bioelectrical impedance; %BF_DXA_: body fat estimated with dual-energy X-ray absorptiometry.

**Table 3:** Correlation between existing anthropometric equations and DXA-derived estimates of assessing body fat percentage in male athletes from combat sports.

Anthropometric vs. DXA	*r*	*p*
Stewart et al.	0.876^∗∗^	<0.001
Civar et al.	0.834^∗∗^	<0.001
Reilly et al.	0.899^∗∗^	<0.001
Oliver et al.	0.907^∗∗^	<0.001
Evans et al. 2	0.907^∗∗^	<0.001
Evans et al. 1	0.905^∗∗^	<0.001
Withers et al.	0.890^∗∗^	<0.001
Thorland et al. 2	0.840^∗∗^	<0.001
Thorland et al. 1	0.906^∗∗^	<0.001
White et al.	0.887^∗∗^	<0.001
Forsyth and Sinning 4	0.886^∗∗^	<0.001
Forsyth and Sinning 3	0.852^∗∗^	<0.001
Forsyth and Sinning 2	0.877^∗∗^	<0.001
Forsyth and Sinning 1	0.848^∗∗^	<0.001
Zuti and Golding	0.569^∗∗^	<0.001
Faulkner	0.904^∗∗^	<0.001
Yuhasz	0.909^∗∗^	<0.001

**Table 4:** Median values of body fat percentages measured with DXA and BIA and estimated by anthropometric equations.

Method	Median (25^th^-75^th^ percentile)
DXA	15.80 (12.70-19.45)
BIA	10.50 (7.45-13.35)
Stewart et al.	10.50 (6.95-15.80)
Civar et al.	13.00 (10.85-16.65)
Reilly et al.	11.60 (10.10-13.90)
Oliver et al.	12.70 (10.55-16.35)
Evans et al. 2	10.90 (8.90-14.25)
Evans et al. 1	10.80 (8.85-14.30)
Withers et al.	13.5 (11.00-17.05)
Thorland et al. 2	9.40 (6.60-12.25)
Thorland et al. 1	11.30 (7.90-16.80)
White et al.	9.70 (7.25-12.60)
Forsyth and Sinning 4	11.90 (8.40-18.05)
Forsyth and Sinning 3	11.80 (8.80-18.50)
Forsyth and Sinning 2	12.00 (8.30-19.25)
Forsyth and Sinning 1	11.80 (8.40-19.10)
Zuti and Golding	18.00 (15.45-21.35)
Faulkner	12.50 (10.80-14.80)
Yuhasz	18.00 (15.45-21.35)

BIA: bioelectrical impedance; DXA: dual-energy X-ray absorptiometry; *r*: Spearman's rank correlation coefficient; *p*: statistical significance; ^∗∗^*p* < 0.001.

The article "Body Fat Evaluation in Male Athletes from Combat Sports by Comparing Anthropometric, Bioimpedance, and Dual-Energy X-Ray Absorptiometry Measurements" was published in 2022. Journal: Biomed Res Int.

**Table 5:** Correlation between BIA and DXA-derived estimates of body fat percentage in male athletes from combat sports.

Methods	*r*	*p*
BIA vs. DXA	0.710^∗∗^	<0.001

BIA: bioelectrical impedance; DXA: dual-energy X-ray absorptiometry; *r*_*s*_: Spearman's rank correlation coefficient; *p*: statistical significance; ^∗∗^*p* < 0.001.

## Data Availability

The data (anthropometric, BIA, and DXA measurements compiled in Excel file, SPSS database, and readings from BIA and DXA scanner) used to support the findings of this study are available from the corresponding author upon request.

## References

[1] Ackland T. R., Lohman T. G., Sundgot-Borgen J. (2012). Current status of body composition assessment in sport. *Sports Medicine*.

[2] Harvey I., Boudreau A., Stephens J. M. (2020). Adipose tissue in health and disease. *Open Biology*.

[3] Kershaw E. E., Flier J. S. (2004). Adipose tissue as an endocrine organ. *The Journal of Clinical Endocrinology and Metabolism*.

[4] Sundgot-Borgen J., Meyer N. L., Lohman T. G. (2013). How to minimise the health risks to athletes who compete in weight-sensitive sports review and position statement on behalf of the ad hoc research working group on body composition, health and performance, under the auspices of the IOC medical commission. *British Journal of Sports Medicine*.

[5] Gabbett T. (2005). Science of rugby league football: a review. *Journal of Sports Sciences*.

[6] Guh D. P., Zhang W., Bansback N., Amarsi Z., Birmingham C. L., Anis A. H. (2009). The incidence of co-morbidities related to obesity and overweight: a systematic review and meta-analysis. *BMC Public Health*.

[7] Silva M. R., Paiva T. (2015). Low energy availability and low body fat of female gymnasts before an international competition. *European Journal of Sport Science*.

[8] Duren D. L., Sherwood R. J., Czerwinski S. A. (2008). Body composition methods: comparisons and interpretation. *Journal of Diabetes Science and Technology*.

The article "Body Fat Evaluation in Male Athletes from Combat Sports by Comparing Anthropometric, Bioimpedance, and Dual-Energy X-Ray Absorptiometry Measurements" was published in 2022. Journal: Biomed Res Int.

[9] Forsyth H. L., Sinning W. E. (1973). The anthropometric estimation of body density and lean body weight of male athletes. *Medicine and Science in Sports*.

[10] Oliver J. M., Lambert B. S., Martin S. E., Green J. S., Crouse S. F. (2012). Predicting football players' dual-energy x-ray absorptiometry body composition using standard anthropometric measures. *Journal of Athletic Training*.

[11] White J., Mayhew J. L., Piper F. C. (1980). Prediction of body composition in college football players. *The Journal of Sports Medicine and Physical Fitness*.

[12] Swann C., Moran A., Piggott D. (2015). Defining elite athletes: issues in the study of expert performance in sport psychology. *Psychology of Sport and Exercise*.

[13] Stewart A., Marfell-Jones M., Olds T., De Ridder H. (2011). International standards for anthropometric assessment. *International Society for the Advancement of Kinanthropometry*.

[14] Yuhasz M. (1962). *The Effects of Sports Training on Body Fat in Man with Predictions of Optimal Body Weight*.

[15] Zuti W. B., Golding L. A. (1973). Equations for estimating percent fat and body density of active adult males. *Medicine and Science in Sports*.

[16] Thorland W. G., Johnson G. O., Tharp G. D., Housh T. J., Cisar C. J. (1984). Estimation of body density in adolescent athletes. *Human Biology*.

[17] Reilly T., George K., Marfell-Jones M., Scott M., Sutton L., Wallace J. (2009). How well do skinfold equations predict percent body fat in elite soccer players?. *International Journal of Sports Medicine*.

[18] Faulkner J. A. (1968). *Physiology of swimming and diving*.

[19] Withers R. T., Craig N. P., Bourdon P. C., Norton K. I. (1987). Relative body fat and anthropometric prediction of body density of male athletes. *European Journal of Applied Physiology and Occupational Physiology*.

[20] Evans E. M., Rowe D. A., Misic M. M., Prior B. M., Arngrímsson S. A. (2005). Skinfold prediction equation for athletes developed using a four-component model. *Medicine and Science in Sports and Exercise*.

[21] Civar S., Aktop A., Tercan E., Ozdol Y., Ozer K. (2006). Validity of leg-to-leg bioelectrical impedance measurement in highly active women. *Journal of Strength and Conditioning Research*.

[22] Siri W. E. (1993). Body composition from fluid spaces and density: analysis of methods. *Nutrition*.

[23] Norton K., Kevin Norton R. E. (2018). *Kinanthropometry and Exercise Physiology*.

[24] Dimitrijevic M., Lalovic D., Milovanov D. (2021). Correlation of different anthropometric methods and bioelectric impedance in assessing body fat percentage of professional male athletes. *Serbian Journal of Experimental and Clinical Research*.

The article "Body Fat Evaluation in Male Athletes from Combat Sports by Comparing Anthropometric, Bioimpedance, and Dual-Energy X-Ray Absorptiometry Measurements" was published in 2022. Journal: Biomed Res Int.

[25] Gibson A. L., Wagner D. R., Heyward V. H. (2018). *Advanced Fitness Assessment and Exercise Prescription*.

[26] Hind K., Slater G., Oldroyd B. (2018). Interpretation of dual-energy X-ray absorptiometry-derived body composition change in athletes: a review and recommendations for best practice. *Journal of Clinical Densitometry*.

[27] Hopkins W., Marshall S., Batterham A., Hanin J. (2009). Progressive statistics for studies in sports medicine and exercise science. *Medicine and Science in Sports and Exercise*.

[28] Riyahi-Alam S., Mansournia M. A., Kabirizadeh Y., Mansournia N., Steyerberg E., Kordi R. (2017). Development and validation of a skinfold model for estimation of body density for a safe weight reduction in young Iranian wrestlers. *Sports Health*.

[29] Davidson L. E., Wang J., Thornton J. C. (2011). Predicting fat percent by skinfolds in racial groups: Durnin and Womersley revisited. *Medicine and Science in Sports and Exercise*.

[30] Stewart A. D., Hannan W. J. (2000). Prediction of fat and fat-free mass in male athletes using dual X-ray absorptiometry as the reference method. *Journal of Sports Sciences*.

[31] Demura S., Yamaji S., Goshi F., Kobayashi H., Sato S., Nagasawa Y. (2002). The validity and reliability of relative body fat estimates and the construction of new prediction equations for young Japanese adult males. *Journal of Sports Sciences*.

[32] Eston R. G., Fu F., Fung L. (1995). Validity of conventional anthropometric techniques for predicting body composition in healthy Chinese adults. *British Journal of Sports Medicine*.

[33] Faulkner J. A. (1966). Physiology of swimming. *American Association for Health, Physical Education and Recreation*.

[34] Bilsborough J. C., Greenway K., Opar D., Livingstone S., Cordy J., Coutts A. J. (2014). The accuracy and precision of DXA for assessing body composition in team sport athletes. *Journal of Sports Sciences*.

[35] Paton N. I., Macallan D. C., Jebb S. A., Pazianas M., Griffin G. E. (1995). Dual-energy X-ray absorptiometry results differ between machines. *Lancet*.

